This article has been retracted.

# Prediction and Analysis of Housing Price Based on the Generalized Linear Regression Model

**DOI:** 10.1155/2022/3590224

**Published:** 2022-09-29

**Authors:** Xinshu Li

**Affiliations:** Faculty of Science, University of Melbourne, Melbourne, Victoria 3010, Australia

## Abstract

In order to improve the reliability of housing price prediction and analysis, this article combines the generalized linear regression model to build a real estate price prediction model and analyzes the basic knowledge of data mining. On the basis of this prior knowledge, this article investigates the cluster analysis algorithm and selects the generalized linear regression model as the research focus based on its definition and the characteristics of stock data. Moreover, this article analyzes the estimation methods of the generalized linear regression model and the nonparametric regression model, and then gives the estimation method of a partial linear model. In addition, this article verifies the validity of the model proposed in this article by means of simulation research. Through the simulation and comparison experiments, it can be seen that the housing price prediction system based on the generalized regression model proposed in this article has a high housing price prediction accuracy.

## 1. Introduction

Nowadays, many people invest in real estate, because sometimes, it can bring a lot of capital income, which has developed very violently in our country. Investment in real estate is also a reflection of a local real estate development situation to a certain extent. For example, if investment is hot, it means that the development is unbalanced, and the supply is in short supply. If investment is cold, it means that the recent real estate market is relatively stable. Moreover, it is also a reflection of the development of a city [1]. However, it does not mean that the more the investment, the better the real estate will develop, the more benefits the investors will get, and there may be negative situations, and some places have suffered from this situation. Moreover, real estate investment in many places has gone wrong, exceeding demand. This is a waste of resources and irresponsible for people's lives, and there will also be situations where workers are not paid, causing social chaos [2]. Therefore, in order to prevent these situations from happening, it is very important to control the investment in real estate. In the process of urbanization, the government should actively formulate reasonable measures to control the situation and ensure that the proportion of investment in fixed assets remains around 25%. Moreover, this limit is not fixed. It also depends on the development of the city. After the initial stage of urban development, this ratio can be appropriately reduced, because there is no need for so many houses at this time [3]. What we need to know very clearly is that we cannot make reasonable improvement measures in a timely manner. The reason for this is that we always know the problem after the situation arises, and it has a certain lag effect. Therefore, when formulating, it is necessary to fully and comprehensively consider the development situation and changes in the relationship between supply and demand, strive to achieve standards that can meet the long-term development situation, and try to avoid the rise in housing prices due to incorrect measures. This is not only a guarantee for the stable development of society, but also a guarantee for people's lives. Only when people are stable can a country develop well [4].

At present, the methods of housing price forecasting can be divided into two categories. One is a multifactor analysis model based on the analysis of the influencing factors of housing prices, and the other is a single-factor analysis based on time series. In the multivariate analysis models, most of them only consider the parameters that affect housing prices, such as multiple regression models, but do not consider the nonparametric factors. The absence of some nonparametric influencing factors is likely to lead to a decrease in the accuracy of the prediction model [5]. In the process of reviewing the literature, only one paper was found that used a partial linear model to predict the average sales price of commercial housing across the country, and the results of the paper showed that the partial linear model was better than the linear regression model in predicting housing prices. This is because the partial linear model considers both linear and nonlinear factors affecting housing prices [6]. However, considering that there are many factors affecting housing prices, there will be a curse of dimensionality when using a partial linear model. The additive model can eliminate the disaster of dimensionality, so it is of great practical significance to build a housing price prediction model based on the additive model. In addition, it also has important theoretical significance to establish a housing price prediction model on the basis of the additive model [7]. In different places, housing prices are affected by local policies and special events, and the fluctuation laws of housing prices are also different.

The definition of real estate in economics is mainly divided into narrow sense and broad sense. Real estate in the broad sense is understood as the sum of real estate commodity relations generated in the exchange process [8]; real estate in the narrow sense is understood as a place used for real estate rental, sale, mortgage, and other commodity transactions [9]. It is worth mentioning that the real estate price in this article is both an equilibrium price and a market price [10].

In the real estate market, consumers refer to buyers, suppliers refer to real estate developers, and the equilibrium price refers to the equilibrium price between the quantity of a certain type of real estate provided by real estate developers. Real estate usually cannot play its role as a commodity independently, and its main value is reflected in its use, which is a kind of induced demand [11].

As a commodity, real estate conforms to the relationship between supply and price in economic theory, but the real estate itself has a large investment scale, a long construction period, and the visibility of recoverable interest rates is longer than that of general commodity cycles. Generally speaking, when the supply of real estate increases, housing prices will rise, which is a positive relationship. However, the entire process of real estate supply is relatively long, and it will have an informatization impact on the market during the construction period, such as investment in real estate. Elements such as quantity, real estate development, and related infrastructure construction will enter the market in the form of information, thereby affecting the judgment and analysis of various market players, and then affecting the changes in real estate prices [12]. However, the effect of this influence path is relatively slow, and the price changes are relatively lag, and the lag time is positively correlated with the risk it brings. The lag time here refers to the time that changes in the supply of real estate act on prices. For developers, the greater the risk, the less incentive they have to develop real estate, the smaller the quantity of real estate provided, the insufficient supply to meet the demand, and the price rise; on the contrary, when the information is more comprehensive and the uncertainty is less, the lower the risk, the greater the motivation for real estate developers to develop, the supply exceeds the demand, and the price decreases [13].

Whether it is a house buyer or a real estate developer, they will make a psychological assessment of the future economic situation when making decisions. This is mainly because people are uncertain about the risks they will face in the future, and an early warning mechanism will be generated in advance. In economics, anticipation is defined as a psychological effect, which refers to the expected effect that people will collect, analyze, and judge before making economic decisions [14]. The real estate market is of great significance in my country and has always been the focus of all sectors of society. However, the information people have is limited, and it is impossible to effectively predict the future real estate market trends and avoid the impact of the economic environment on real estate. Therefore, expectations are correct. Both the buyer and the real estate developer are very important. For home buyers, they will have a rough expectation of future house prices based on the current and future real estate market conditions, as well as the trend of real estate prices in the past period of time. If the real estate price is on an upward trend in the future, then the demand for housing will also increase whether it is for consumption demand or investment demand [15]; if the real estate price is on a downward trend in the future, then demand will also drop. In addition, the surrounding supporting equipment of real estate also affects the psychological expectations of home buyers, including traffic conditions, infrastructure construction, and green area, especially schools, hospitals, and other factors [16].

This article uses the generalized linear regression model to construct the real estate price prediction model, verifies the validity of the model in this article by comparing the actual data and simulation research, and promotes the accuracy of subsequent real estate price prediction.

## 2. Generalized Linear Regression Prediction

### 2.1. Cluster Analysis

Data similarity refers to the calculation method of similarity between data objects. There are generally two methods to describe the similarity between data objects: one is the distance, and the other is the similarity coefficient. The so-called distance refers to depicting the distance between objects according to the relationship between close and distant, that is, putting the closest ones together and combining them into one class. The similarity coefficient is a numerical value between 0 and 1, indicating the similarity between the two. When the similarity coefficient is closer to 1, the similarity between the two is greater; when the similarity coefficient is closer to 0, the similarity between the two is smaller. Cluster analysis is often divided into R-type clustering and *Q*-type clustering. Among them, the *R*-type clustering often uses the correlation coefficient to describe the similarity, and the *Q*-type clustering often uses the distance measurement to describe the similarity.

#### 2.1.1. Two Categorical Variables

For binary variables, the similarity matrix is used to describe the similarity between objects, and it considers observations (*x*_*i*_, *x*_*j*_), where *x*_*i*_^*T*^=(*x*_*i*1_, *x*_*i*2_, ⋯, *x*_ip_), *x*_*j*_^*T*^=(*x*_*j*1_, *x*_*j*2_, ⋯, *x*_jp_) and *x*_*ik*_, *x*_*jk*_ ∈ {0,1}.

Among them, there exists *a*_*t*_, *t*=1,2,3,4, and its value depends on the pair (*x*_*i*_, *x*_*j*_). Therefore, the similarity characterization formula used in daily life can be given as

(1) $$\begin{array}{c} d_{ij}=\frac{a_{1}+\delta a_{4}}{a_{1}+\delta a_{4}+\lambda \left(a_{2}+a_{3}\right)}\text{,} \end{array}$$

where *δ*, *λ* is the weight coefficient.

#### 2.1.2. Continuous Variables

*(1) Numerical Continuous Variables*. The following formula is defined as

(2) $$\begin{array}{c} d_{ij}=\left\|x_{i}-x_{j}\right\|={\left(\overset{n}{\underset{k=1}{\sum }}{\left|x_{ik}-x_{jk}\right|}^{r}\right)}^{1/r}\text{,} \end{array}$$

where *x*_*ik*_ represents the *k*th attribute value of the *i*th object, *d*_*ii*_=0, ∀*i*=1,2, ⋯, *n*.

When *r* = 1, the above formula is the absolute distance; when *r* = 2, the above formula is the Euclidean distance; when *r*=*∞*, the above formula is the Chebyshev distance.

*(2) Vector-Type Continuous Variable*. If we encounter numerical variables that are not on the same metric, we first need to standardize them, so we introduce a more general metric—Mahalanobis distance, where the data object is in the form of a vector:

(3) $$\begin{array}{c} d=\left(x-y\right)\overset{-1}{\sum }{\left(x-y\right)}^{T}\text{.} \end{array}$$

The similarity coefficient is a numerical value between 0 and 1, indicating the similarity between the two. The similarity between the two is smaller. In the following, a few commonly used formulas are introduced:

(1) Exponential similarity coefficient formula
  (4) $$\begin{array}{c} r_{ij}=\frac{1}{m}\overset{m}{\underset{k=1}{\sum }}\exp\left[-\frac{3}{4}\frac{{\left(x_{ij}-x_{jk}\right)}^{2}}{s_{k}^{2}}\right]\left(i,j=1,2,\cdots ,n\right), \end{array}$$
  (5) $$\begin{array}{c} s_{k}={\left[\frac{1}{n}\overset{n}{\underset{i=1}{\sum }}{\left(x_{ik}-{\bar{x}}_{k}\right)}^{2}\right]}^{\left(1/2\right)}k=\left(1,2,\cdots ,m\right),\\ {\bar{x}}_{k}=\frac{1}{n}\overset{n}{\underset{i=1}{\sum }}x_{ik}k=\left(1,2,\cdots ,m\right). \end{array}$$
(2) Cosine formula of the included angle
  (6) $$\begin{array}{c} r_{ij}=\frac{\left|\sum_{k=1}^{m}x_{ik}x_{ik}\right|}{{\left[\sum_{k=1}^{m}x_{ik}^{2}\sum_{k=1}^{m}x_{jk}^{2}\right]}^{\left(1/2\right)}},\left(i,j=1,2,\cdots ,n\right)\text{.} \end{array}$$
(3) Correlation coefficient formula
  (7) $$\begin{array}{c} r_{ij}=\frac{\left|\sum_{k=1}^{m}\left(x_{ik}-{\bar{x}}_{i}\right)\left(x_{jk}-{\bar{x}}_{j}\right)\right|}{{\left[\sum_{k=1}^{m}{\left(x_{ik}-{\bar{x}}_{i}\right)}^{2}\overset{m}{\underset{k=1}{\sum }}{\left(x_{jk}-{\bar{x}}_{j}\right)}^{2}\right]}^{\left(1/2\right)}},\left(i,j=1,2,\cdots ,n\right), \end{array}$$

where ${\bar{x}}_{i}=\left(1/m\right)\sum_{k=1}^{m}x_{ik};{\bar{x}}_{j}=\left(1/m\right)\sum_{k=1}^{m}x_{jk}$.

The algorithm flow is as follows: first, the algorithm needs to determine the number of cluster categories *k* and perform initial clustering on the dataset.

The algorithm steps are as follows:

(1) The algorithm selects *k* initial clustering centers: *z*_1_^(1)^, *z*_2_^(1)^, ⋯, *z*_*k*_^(1)^, where the superscript indicates the number of iterative operations in the clustering process.
(2) When the rth iteration has been performed, if for a certain sample *x*, there is
  (8) $$\begin{array}{c} d\left(x,z_{j}^{\left(r\right)}\right)=\min\;\left\{d\left(x,z_{i}^{\left(r\right)}\right),i=1,2,\cdots ,k\right\}, \end{array}$$
then, *x* ∈ *S*_*j*_^(*r*)^.*S*_*j*_^(*r*)^ is a subset of samples with *z*_*j*_^(*r*)^ as the cluster center. In this way, that is, the principle of minimum distance, all samples are assigned to *k* cluster centers.
(3) The algorithm calculates the reclassified cluster centers:
  (9) $$\begin{array}{c} z_{j}^{\left(r+1\right)}=\frac{1}{n_{j}^{\left(r\right)}}\underset{x\in S_{j}^{\left(r\right)}}{\sum }x,\left(j=1,2,\cdots K\right), \end{array}$$
where *n*_*j*_^(*r*)^ is the number of samples included in *S*_*j*_^(*r*)^.
(4) If *z*_*i*_^(*r*+1)^=*z*_*j*_^(*r*)^, *j*=1,2, ⋯*K*, the algorithm ends; otherwise, the algorithm goes to (2).

### 2.2. Random Process

Such a random process is called a Markov chain, if it takes only a finite or listable number of values, and for any *Q* and any state *W*, we have

(10) $$\begin{array}{c} P\left\{X_{n+1}=j|X_{n}=i,X_{n-1}=i_{n-1},\cdots ,X_{1}=i_{1},X_{0}=i_{0}\right\}\\ =P\left\{X_{n+1}=j|X_{n}=i\right\}\\ =P_{ij}, \end{array}$$

where *X*_*n*_=*i* indicates that the process is in state *i* at time *n*, and {0,1,2, ⋯} is called the state space of the process, denoted as *S*. The above formula describes the characteristics of the Markov chain, which is called the Markov property. When given the past states *X*_0_, *X*_1_, ⋯, *X*_*n*−1_ and the present state *X*_*n*_|, the conditional distribution of the future state *X*_*n*+1_ is independent of the past state and only depends on the present state. That is to say, the Markov chain has no aftereffect. We also conduct research on housing prices based on the ineffectiveness of Markov chains.

The conditional probability *P*_*ij*_=*P*{*X*_*n*+1_=*j|X*_*n*_=*i*} is the one-step transition probability of the Markov chain {*X*_*n*_, *n*=0,1,2, ⋯}, referred to as the transition probability, denoted as *P*_*ij*_. It represents the probability of being in state *i* and moving to state *j* next. When the transition probability *Q* = 1 of the Markov chain is only related to the states *i*, *j*, and it has nothing to do with *n*, it is called a time-aligned Markov chain. Otherwise, it is called a non-time-aligned chain. The transition probability matrix is given as

(11) $$\begin{array}{c} P=\left(p_{ij}\right)=\left[\begin{array}{cccc} p_{00} & p_{01} & \cdots & p_{0,N-1}\\ p_{10} & p_{11} & \cdots & p_{1,N-1}\\ \vdots & \vdots & \vdots & \vdots \\ p_{N-1,0} & p_{N-1,1} & \cdots & p_{N-1,N-1} \end{array}\right], \end{array}$$

where *P* is called the transition probability matrix, generally referred to as the transition matrix. Since the probability is non-negative and the process must transition to some state, it is easy to see that *p*_*ij*_(*i*, *j* ∈ *S*) has the following properties:

1. *p*_*ij*_ ≥ 0, *ij* ∈ *S*;
2. ∑*p*_ij_=1, ∀*i* ∈ *S*.

In practical applications, the one-step transition probability is generally difficult to obtain directly, and the method of using frequency instead of probability is often considered to count the number of transitions *m*_ij_ from a fixed state *i* to other states *j*, and count the total number of times in state *i*. Therefore, we get *p*_*ij*_=(*m*_*ij*_/*m*_*i*_).

The *n*-step transition probability is called the conditional probability:

(12) $$\begin{array}{c} p_{ij}^{\left(n\right)}=P\left(X_{m+n}=j|X_{m}=i\right),i,j\in S;m\geq 0;n\geq 1. \end{array}$$

It is the n-step transition probability of the Markov chain, and correspondingly, *P*^(*n*)^=(*p*_*ij*_^(*n*)^) is called the n-step transition probability matrix. When *n* = 1, *p*_*ij*_^(1)^=*p*_*ij*_, *P*^(1)^=*P*. In addition, it stipulates

(13) $$\begin{array}{c} p_{ij}^{\left(0\right)}=\left\{\begin{array}{cc} 0\text{,} & i\neq j\text{,}\\ 1\text{,} & i=j\text{.} \end{array}\right. \end{array}$$

It has nothing to do with the state that the intermediate n-1 steps transition through.

Classification and nature of states:

(1) Irreducible Markov chain
State *i* is said to be reachable to state j(*i*, *j* ∈ *S*), and if there exists *n* ≥ 0 such that p_*i*j_^*n*^ > 0.
We classify any two intercommunication states into a class, the states in the same class should all be intercommunicated, and any state cannot belong to two different classes at the same time.
From this, we can get the definition of irreducible Markov chain.
Moreover, it is specially stipulated that when the abovementioned set is an empty set, the period of *i* is said to be infinite.
(2) Always return state.
For any state *i,j*, *f*_*ij*_^(*n*)^ is the probability of reaching *j* for the first time from *i* after *n* steps, and obviously, *f*_*ij*_=∑_*n*=1_^*∞*^*f*_*ij*_^(*n*)^. If *f*_*ij*_=1, state *j* is said to be a constant return state. If *f*_ij_ < 1, the state *j* is said to be a nonrecurrent state or an instantaneous state.
For the constant return state *i*, *u*_*i*_ represents the average number of steps (time) required to start from *i* and then return to *i*, as shown in the following formula:
  (14) $$\begin{array}{c} u_{i}=\overset{\infty }{\underset{n=1}{\sum }}nf_{ii}^{\left(n\right)}. \end{array}$$

Among them, if *u*_*i*_ < +*∞*, then *i* is called the normal return state. If *u*_*i*_=+*∞*, then *i* is called the zero return state. If *i* is a normal return state and is aperiodic, it is called an ergodic state. If *i* is an ergodic state and *f*_*ii*_^(1)^=1, *i* is called an absorbing state, and obviously *u*_*i*_=1.

For an irreducible aperiodic Markov chain, if it is ergodic, then $\pi_{j}=\lim_{n⟶\infty }p_{ij}^{\left(n\right)}>0\left(j\in S\right)$ is a stationary distribution and the only stationary distribution. A stationary distribution does not exist if the states are all instantaneous or all zeros are recurring. The stationary distribution satisfies the following formula:

(15) $$\begin{array}{c} \left\{\begin{array}{c} \underset{j\in S}{\sum }\pi_{j}=1\\ \underset{i\in S}{\sum }\pi_{i}p_{ij}^{\left(n\right)}=\pi_{j}. \end{array}\right. \end{array}$$

For the traversed Markov chain, if all states are connected and are normal return states with period 1, the limit is given as

(16) $$\begin{array}{c} \lim_{n⟶\infty i}p_{ij}^{\left(n\right)}=\pi_{j},j\in S. \end{array}$$

It is called the limit distribution of the Markov chain, that is, *π*_*j*_=(1/*u*_*j*_). The limiting distribution is the stationary distribution and the only stationary distribution.

#### 2.2.1. Calculation of the One-Step Transition Probability Matrix

In practical applications, it is generally difficult to directly obtain the one-step transition probability, so the method of using frequency instead of probability is often considered.

First, the frequency transition matrix *M* is obtained, that is, to count the number *m*_*ij*_ of transitions from a fixed state *i* to other states *j*:

(17) $$\begin{array}{c} M=\left[\begin{array}{cccc} m_{00} & m_{01} & \cdots & m_{0,N-1}\\ m_{10} & m_{11} & \cdots & m_{1,N-1}\\ \vdots & \vdots & \vdots & \vdots \\ m_{N-1,0} & m_{N-1,1} & \cdots & m_{N-1,N-1} \end{array}\right]\text{.} \end{array}$$

Then, the total number of times in state *i* is counted, which is calculated according to the following formula:

(18) $$\begin{array}{c} p_{ij}=\left\{\begin{array}{cc} \frac{m_{ij}}{\sum_{j\in S}m_{ij}} & \sum_{j\in S}m_{ij}>0,\\ 0 & \sum_{j\in S}m_{ij}=0, \end{array}\right. \end{array}$$

where *m*_*i*_=∑_*j*=0_^*N*^*m*_*ij*_

Finally, the transition probability matrix P is calculated, that is, the probability is replaced by frequency:

(19) $$\begin{array}{c} P=\left[\begin{array}{cccc} p_{00} & p_{01} & \cdots & p_{0,N-1}\\ p_{10} & p_{11} & \cdots & p_{1,N-1}\\ \vdots & \vdots & \vdots & \vdots \\ p_{N-1,0} & p_{N-1,1} & \cdots & p_{N-1,N-1} \end{array}\right]\text{.} \end{array}$$

#### 2.2.2. Markov Test

Before using the Markov chain to build a prediction model, the Markov property of the sequence {*X*_*t*_, *t* ∈ *T*} must be checked. The test is performed using the *χ*^2^ statistic.

Test statistics:

(20) $$\begin{array}{c} {\hat{\chi }}^{2}=2\overset{m}{\underset{i=1}{\sum }}\overset{m}{\underset{j=i}{\sum }}n_{ij}\left|\log\left(\frac{P_{ij}}{{\hat{P}}_{.j}}\right)\right|, \end{array}$$

where ${\hat{P}}_{.j}=\sum_{i=1}^{m}n_{ij}/\sum_{i=1}^{m}\sum_{k=1}^{m}n_{ik}an\;d\;P_{ij}=n_{ij}/\sum_{k=1}^{m}n_{ik}$. When *m* is larger, the above obeys the chi-square distribution, and the degree of freedom is (*m* − 1)^2^.

The confidence level *α* is chosen. If the statistic is ${\hat{\chi }}^{2}>\chi_{\alpha }^{2}{\left(m-1\right)}^{2}$, then the null hypothesis is rejected, and the sequence {*X*_*t*_, *t* ∈ *T*} is considered to be Markov's, and the model can be used to make predictions after passing the Markov test, and vice versa.

#### 2.2.3. Stable Distribution

From the transition probability matrix, a stationary distribution *π*_*j*_ is derived.

(21) $$\begin{array}{c} \left\{\begin{array}{c} \underset{j\in S}{\sum }\pi_{j}=1,\\ \underset{i\in S}{\sum }\pi_{i}p_{ij}^{\left(n\right)}=\pi_{j}. \end{array}\right. \end{array}$$

#### 2.2.4. Making Predictions Based on the Initial State

It is known that the initial state is *x*_0_, and if it is in state *i*, then *x*_0_=(0, ⋯, 0,1,0, ⋯0), that is, the probability of being in state *i* at this time is 1, and the rest are 0.

(22) $$\begin{array}{c} x_{1}=x_{0}*p. \end{array}$$

The state of the system at time *t* + 1 can be obtained.

We set *x*_1_=(*x*_1_^(1)^, *x*_1_^(2)^, ⋯, *x*_1_^(*n*)^). According to the principle of maximization, we can get

(23) $$\begin{array}{c} \max\;\left\{\left(x_{1}^{\left(1\right)},x_{1}^{\left(2\right)},\cdots ,x_{1}^{\left(n\right)}\right)\right\}=x_{1}^{\left(j\right)}. \end{array}$$

Therefore, the next moment is most likely to be in state *j*.

### 2.3. Time Series Analysis

#### 2.3.1. Stationary Time Series

Stationary time series mean and variance do not change systematically and do not change periodically. Each observation value in this type of series basically fluctuates at a fixed level. Although the degree of fluctuation is different in different time periods, there is no certain rule, and its fluctuation can be regarded as random. Stationary distribution includes general autoregressive model AR(*p*), moving average model MA(*q*), and autoregressive moving average model ARMA(*p*, *q*).

An autoregressive model is a process of using itself as a regression variable, that is, a linear regression model that uses the linear combination of random variables at several previous moments to describe random variables at a certain time in the future. It is a common form in time series.

Consider a time series *y*_1_, *y*_2_, ⋯, *y*_*n*_, *p*-order autoregressive model (abbreviated AR(*p*)) indicating that *Z* in the series is a linear combination of the first *p* series and a function of the error term; the general form of the mathematical model is

(24) $$\begin{array}{c} y_{t}=\alpha_{1}y_{t-1}+\alpha_{2}y_{t-2}+\cdots +\alpha_{p}y_{t-p}+\omega_{t,} \end{array}$$

where *p* is called the order of the autoregressive model, denoted as AR(*p*). *α*_1_, ⋯, *α*_*p*_ is the model parameter, *ω*_*t*_ is white noise with mean 0 and variance *σ*^2^.

There are similarities between moving average MA(*q*) models and autoregressive models.

If a univariate time series data is {*y*_*t*_; *t*=1,2, ⋯},

(25) $$\begin{array}{c} y_{t}=\omega_{t}+\beta_{1}\omega_{t-1}+\cdots +\beta_{p}\omega_{t-p}. \end{array}$$

AR models are attempts to capture and explain the momentum and mean reversal effects of financial trading markets. The MA model is an attempt to capture and explain the observed oscillatory effects in the white noise term, which can be understood as the effects of unintended events that affect the observed process.

The ARMA model is a combination of the two. Its main disadvantage is that it ignores the fluctuation clustering phenomenon often seen in financial market time series data. The model formula is as follows:

(26) $$\begin{array}{c} y_{t}=\alpha_{1}y_{t-1}+\alpha_{2}y_{t-2}+\cdots +\alpha_{p}y_{t-p}+\omega_{t}+\beta_{1}\omega_{t-1}+\cdots +\beta_{q}\omega_{t-q}\\ =\overset{p}{\underset{i=1}{\sum }}\alpha_{i}y_{t-i}+\omega_{t}+\overset{q}{\underset{i=1}{\sum }}\beta_{i}\omega_{t-i}. \end{array}$$

#### 2.3.2. Nonstationary Time Series

Nonstationary distributions include (*p*, *d*, *q*).

Finally, the ARIMA model is used as a comparative model to highlight the accuracy and practicability of the model built in this subject.  Figure 1 shows the specific modeling steps.

If the sequence is nonstationary, it can be made stationary with the help of difference operation. Nonstationary series can be written as

(27) $$\begin{array}{c} X_{t}=\mu_{t}+\xi_{t}=\overset{d}{\underset{j=0}{\sum }}\beta_{j}t^{j}+\Theta \left(B\right)\varepsilon_{t}. \end{array}$$

Among them, {*ε*_*t*_} is a white noise sequence with zero mean.

For example, the first difference is

(28) $$\begin{array}{c} \nabla X_{t}=X_{t}-X_{t-1}. \end{array}$$

The formula for calculation is as follows:

(29) $$\begin{array}{c} ACF\left(k\right)=\rho_{k}=\frac{cov\left(y_{t},y_{t-k}\right)}{Var\left(y_{t}\right)}, \end{array}$$

where *k* represents the number of lag periods.

The determination of the *p*, *q*-order of the ARIMA(*p,d,q*) model is determined by ACF and PACF, as shown in Table 1.

Null hypothesis: the residual sequence is a white noise sequence.

(30) $$\begin{array}{c} H_{0}:\rho_{1}=\rho_{2}=\cdots =\rho_{m}=0,\forall m\geq 1. \end{array}$$

Alternative hypothesis: the residual sequence is a nonwhite noise sequence.

*H*_1_: there is at least one *ρ*_*k*_ ≠ 0, ∀*m* ≥ 1, *k* ≤ *m*

Test statistics:

(31) $$\begin{array}{c} LB=N\left(N+2\right)\overset{m}{\underset{k=1}{\sum }}\frac{{\hat{\rho }}_{k}^{2}}{N-K}∼\chi^{2}\left(m\right). \end{array}$$

If the test result is to reject the null hypothesis, it means that the residual sequence is a nonwhite noise sequence, and the useful information in the residual sequence has not been fully extracted. It further shows that the fitted model is not significant. If the residual sequence is a white noise sequence, the null hypothesis is not rejected, indicating that the fitted model is significantly effective.

## 3. Prediction and Analysis of Housing Price Based on Generalized Linear Regression Model

Due to the duality of real estate, it can not only provide services for households as consumption, but also provide assets for households as investment. Therefore, the real estate market can be regarded as consisting of three submarkets that interact with each other: the real estate use market, the real estate asset holding market, and the real estate production market. According to their interrelationships, a four-quadrant model is constructed using the rectangular coordinate quadrants, as shown in Figure 2.

Based on the idea of The Economic Cycle Cube, a cube of influencing factors of urban real estate prices is constructed, as shown in Figure 3.

A heterogeneous commodity has different characteristics that meet the needs of consumers, and the implicit price of these heterogeneous characteristics can be calculated by regression, as shown in Figure 4.

Based on the theory of supply and demand, this article divides the participants in the real estate market into real estate developers and home buyers, and divides their behavior into three stages, as shown in Figure 5.

In terms of keyword selection and network information crawling processing, this article mainly adopts the technical means of machine learning, as shown in Figure 6.

According to the established partial linear model, the fitting result of the model is calculated and compared with the real value of the average sales price of commercial housing, and the two curves are drawn, as shown in Figure 7.

It can be seen that the fitted value is relatively close to the real value, and the fitting curve and the real curve have the same trend of change, and the simulation effect is good. The scatter plots of the error term and the two principal components (GDP (100 million yuan) and urban population (10,000 people)) are made, respectively, as shown in Figures 8(a) and 8(b).

According to the established linear regression model, the fitting result of the model is calculated and compared with the real value of the average sales price of commercial housing, and the two curves are drawn, as shown in Figure 9(a). In order to compare the fitting results of the partial linear model and the linear regression model more clearly, we draw the real curve of the national average sales price of commercial housing, the fitted curve of the partial linear model, and the fitted curve of the linear regression model in one graph, as shown in Figure 9(b).

It can be seen from the above research that the housing price prediction system based on the generalized regression model proposed in this article has a high housing price prediction accuracy.

## 4. Conclusion

The demand for commercial housing is generally divided into self-occupied demand, investment demand, and speculative demand. Self-occupation demand is self-occupation; investment demand is to buy commercial housing and rent it out to obtain rental income; speculative demand buys commercial housing in anticipation of rising house prices and sells it after the price rises; and the purpose is to earn the price difference. The demand for self-occupation and investment is the supporting force of the commercial housing market. In particular, the demand for self-occupation has been encouraged and supported by policies. In addition to driving up housing prices, speculative demand squeezes out part of the demand for owner-occupiers and blows up the housing market bubble, which is harmful to the commercial housing market. This article combines the generalized linear regression model to build a real estate price prediction model. Through the simulation and comparison experiments, it can be seen that the housing price forecasting system based on the generalized regression model proposed in this article has a high housing price forecasting accuracy.

## Figures and Tables

**Figure 1:** Flowchart of ARIMA modeling steps.

**Figure 2:** Four-quadrant equilibrium diagram of the real estate market.

**Figure 3:** Cube of influencing factors of urban real estate prices.

**Figure 4:** Equilibrium process of house price in the hedonic price model.

**Figure 5:** Conceptual framework.

**Figure 6:** Technical framework.

**Figure 7:** The real curve of the national average sales price of commercial housing and the fitted curve simulated by a partial linear model.

**Figure 8:** Scatter plot of error terms and principal components. (a) Scatter plot of the error term and the first principal component and (b) scatter plot of the error term and the second principal component.

**Figure 9:** Fitting curve. (a) The real curve of the national average selling price of commercial housing and the fitted curve simulated by a linear regression model and (b) the true curve of the national average sales price of commercial housing and the fitted curve of the two models.

**Table 1:** Determination of *p*, *q*-order.

Model	ACF	PACF
AR(p)	Trailing	*p*-order truncation
MA(q)	*q*-order truncation	Trailing
ARMA()	Trailing	Trailing

## Data Availability

The labeled dataset used to support the findings of this study can be obtained from the corresponding author upon request.
